# Markers of Oxidant-Antioxidant Equilibrium in Patients with Sudden Sensorineural Hearing Loss Treated with Hyperbaric Oxygen Therapy

**DOI:** 10.1155/2019/8472346

**Published:** 2019-02-06

**Authors:** Jarosław Paprocki, Paweł Sutkowy, Jacek Piechocki, Alina Woźniak

**Affiliations:** ^1^Department of Medical Biology and Biochemistry, Collegium Medicum of Nicolaus Copernicus University, Karłowicza 24, 85-092 Bydgoszcz, Poland; ^2^Mazovian Centre for Hyperbaric Therapy and Wound Treatment in Warsaw, Wołoska 137, bud. “O”, 02-507 Warszawa, Poland

## Abstract

The concentration of thiobarbituric acid reactive substances (TBARSs) in plasma and erythrocytes, the activity of selected antioxidant enzymes in erythrocytes: catalase (CAT), superoxide dismutase (SOD), and glutathione peroxidase (GPx), and the levels of hemoglobin (HGB) and haematocrit (HCT) were determined in 40 patients with sudden sensorineural hearing loss (SSNHL) subjected to 14 treatment sessions in a Haux Starmed 2200 hyperbaric chamber. Hyperbaric oxygen (HBO) therapy involved breathing 100% oxygen at 0.25 MPa. Blood for analysis was collected from the basilic vein at three time points: before the first HBO session, approximately 5 min after the first session, and after the 14th session. The control group included 20 healthy individuals never before treated with HBO therapy. Compared to the pre-HBO values, a 10% increase (*P* < 0.05) in the TBARS concentration in erythrocytes, a 28% increase in the GPx activity (*P* < 0.05), and a 7% decrease in the SOD activity (*P* < 0.05) were observed after 14 HBO sessions. The CAT activity decreased by 6% (*P* < 0.05) after the first session. The TBARS concentration in plasma was 13% higher (*P* < 0.01), while that in erythrocytes was 24% lower (*P* < 0.001) in the SSNHL patients before the first HBO session compared to the control group. The CAT activity in the SSNHL patients before HBO therapy was 26% higher (*P* < 0.001) than that in the control group. A statistically significant reduction in HGB and HCT after 14 HBO sessions (*P* < 0.01) compared to the pre-HBO values was demonstrated. SSNHL is accompanied by disturbance in the oxidant-antioxidant equilibrium. Repeated stimulation with hyperbaric oxygen modulates the activity of antioxidant enzymes. It seems that the increased generation of hydrogen peroxide is responsible for the changes in the activity of antioxidant barrier enzymes observed after HBO sessions.

## 1. Introduction

Sudden sensorineural hearing loss (SSNHL) is impairment of the hearing of unknown aetiology, developing over 72 hours. It usually affects one ear, less often both. The age group most frequently affected is people aged 30 to 60 years [1]. The main audiometric criterion of SSNHL is hearing impairment no deeper than 30 dB affecting at least 3 neighbouring frequencies [2, 3]. The incidence of SSNHL in Poland is 5–20 cases per 100,000 people per year [2]. There is no clearly understood cause of this condition, but the most common aetiologies mentioned in the literature include vascular, viral, and autoimmune factors. SSNHL is treated pharmacologically using corticosteroids, antiviral drugs, thrombolytic agents, and vitamins [1]. Hyperbaric oxygen (HBO) therapy, increasingly used by otolaryngologists in treating SSNHL, consists of breathing 100% oxygen in a specially adapted chamber in which the pressure is approximately 2.5 ATA [4]. HBO therapy can be used directly after the occurrence of SSNHL as a primary treatment, alone or together with pharmacotherapy, or as a secondary treatment [2]. In studies, the beneficial effect of this method in treating SSNHL has been associated with improved microcirculation and facilitated diffusion of oxygen from capillary vessels to tissues. After HBO sessions, an increase in the partial pressure of oxygen in the cochlea and reduced hypoxia and oedema of tissues are observed. Moreover, the response to infections and ischaemia in the patient is altered [1].

The purpose of aerobic metabolism is the production of chemical energy stored in ATP, mainly in the process of oxidative phosphorylation [5]. A side effect of this process is the formation of reactive oxygen species (ROS), including oxygen free radicals (OFR), particularly during an incomplete reduction of oxygen in the oxidative chain [5]. The condition in which the generation of ROS exceeds the antioxidant capacity of the body is called oxidative stress [6]. Antioxidant enzymes, such as catalase (CAT), superoxide dismutase (SOD), and glutathione peroxidase (GPx), are responsible for scavenging ROS in the human body [6]. One of the consequences of oxidative stress is increased intensity of lipid peroxidation—free radical chain reactions leading to the oxidation of polyunsaturated fatty acids that form, e.g., cell membranes. Oxidation of polyunsaturated fatty acids leads to the enzymatic or nonenzymatic production of multiple final *α*,*β*-unsaturated aldehyde products, such as malondialdehyde (MDA)—a mutagen commonly used as a biomarker of lipid peroxidation [7]. It has already been seen that HBO increases the production of oxygen free radicals whose effect on the body can be both beneficial and adverse. Therefore, it is possible that this form of therapy induces oxidative stress [8].

The aim of the study was to determine the effect of 14 HBO therapy sessions on the concentration of thiobarbituric acid reactive substances (TBARSs) in plasma and erythrocytes, the activity of key antioxidant enzymes: SOD, CAT, and GPx, and the levels of haemoglobin (HGB) and haematocrit (HCT) in patients with SSNHL.

## 2. Material and Methods

The study was approved by the Bioethics Committee of Ludwik Rydygier Collegium Medicum in Bydgoszcz, Nicolaus Copernicus University, in Torun, Poland (approval no.: KB 260/2016).

### 2.1. Study Subject

The study was conducted in 40 patients (23 men and 17 women; mean age: 43.2 ± 16.0 years) of the Mazovian Centre for Hyperbaric Therapy and Wound Treatment in Warsaw, Poland, treated with HBO therapy for SSNHL. HBO therapy was initiated no later than 5 days after the onset of SSNHL. The patients underwent 14 sessions (conducted daily, one per day) in the hyperbaric chamber, Haux Starmed 2200 used at the Mazovian Centre for Hyperbaric Therapy and Wound Treatment in Warsaw (Figures 1 and 2). The patients received systemic corticosteroidotherapy recommended as the first-line therapy in SSNHL. For the duration of the experiment, the patients were orally administered prednisone (a loading dose of 1 mg/kg of body weight per day, with the usual maximum dose of 60 mg/day) at a gradually tapered dosage until discontinuation. Corticosteroidotherapy was initiated immediately after the diagnosis of SSNHL and continued for 2 weeks. The first and second time points of the study occurred during prednisone therapy, while the third time point occurred after the completion of prednisone therapy. When therapy was completed, an improvement in hearing (within the range of 10–20 dB) was observed in 30 patients.

Participants with other health problems characterised by a proven disruption of the oxidant-antioxidant equilibrium were excluded from the study.

The control group consisted of 20 healthy volunteers (12 men and 8 women; mean age: 28.1 ± 7.1 years) never before treated with HBO therapy.

The employed hyperbaric chamber allowed maintaining equal environmental conditions, i.e., pressure, temperature, and air humidity, and enabled breathing 100% oxygen for the same period for each participant. The inside of the chamber was filled with a breathing gas mixture in which the concentration of oxygen did not exceed 23%, but the study participants breathed 100% oxygen using masks. Hyperbaric oxygen (HBO) therapy involved breathing 100% oxygen at 0.25 MPa. The sessions lasted 90 min and included two 10-minute periods of compression and decompression. Three HBO therapy subsessions, lasting 20 minutes each, were separated by two 5-minute breaks during which the participants breathed the air inside the chamber. Each complete HBO session cycle was as follows: 10 min compression+20 min oxygen therapy+5 min breathing the air inside the chamber+20 min oxygen therapy+5 min breathing the air inside the chamber+20 min oxygen therapy+10 min decompression.

In the SSNHL patients, blood for analysis was collected from the basilic vein at three time points: before the first HBO session, approximately 5 min after the first session, and after the full series of 14 sessions. The biochemical analyses were conducted at a laboratory of biochemistry at the Department of Medical Biology and Biochemistry of the Collegium Medicum of Nicolaus Copernicus University, Poland. In the control group members, blood samples were taken once. The samples were analysed for the concentration of TBARS in erythrocytes and plasma, the activity of CAT, SOD, and GPx in erythrocytes, and the HGB and HCT values.

### 2.2. Methods

The TBARS concentration was determined following a method by Buege and Aust [9] as modified by Esterbauer and Cheeseman [10]. Lipid peroxidation products were identified using thiobarbituric acid (TBA). Malondialdehyde (MDA) is the main but not the only lipid peroxidation product that reacts with TBA. For the sake of simplicity, the level of all substances reacting with TBA was presented as the MDA concentration.

The CAT activity was determined by measuring the decrease in the absorbance of a solution of hydrogen peroxide (H_2_O_2_) decomposed by the enzyme. The decrease in the absorbance value is directly proportional to the reduction of the H_2_O_2_ concentration in the solution [11]. The CAT activity was expressed in IU/g Hb.

The SOD activity was determined based on the inhibition of adrenaline autoxidation to adrenochrome in alkaline conditions. To measure the SOD activity, a previously obtained haemolysate after removal of haemoglobin with a chloroform-ethanol mixture was used. After centrifugation, two layers were obtained: lower layer containing denatured haemoglobin and chloroform and upper layer containing the enzyme [12]. To determine the SOD activity, continuous recording of the reaction was conducted using a reaction kinetics programme on a Varian spectrophotometer. The SOD activity was expressed in U/g Hb.

The GPx activity was determined at 20°C using a method based on the decomposition of hydrogen peroxide by the enzyme with the concurrent oxidation of reduced glutathione [13]. The results were expressed in U/g Hb.

### 2.3. Statistical Analysis

The TBARS concentration in plasma and erythrocytes and the activities of CAT, SOD, and GPx were analysed using the comparative analysis of variance (ANOVA; Tukey's range test) (*STATISTICA v.* 9.1). For the assessment of the statistical significance of the HGB and HCT values measured before the first and after the 14th HBO sessions, Student's *t*-test was used. Differences at significance level *P* < 0.05 were presumed as statistically significant. Dependencies between the analysed parameters were assessed using correlation matrices. A statistical hypothesis of the significance of the correlation coefficients (*r*) was tested.

## 3. Results

The TBARS concentration in the plasma of the SSNHL patients before the HBO therapy was 13% higher than in the healthy members of the control group, and the difference was statistically significant (*P* < 0.01) (Table 1). Approximately 5 min after the first HBO session and then after 14 HBO sessions, the plasma TBARS concentration did not change in a statistically significant manner compared to the that in the pretreatment level and was significantly higher than that in the control group (by 18%, *P* < 0.001, and 11%, *P* < 0.05, respectively).

The TBARS concentration in the erythrocytes of the SSNHL patients before the HBO therapy was 24% lower than that in the control group, and the difference was statistically significant (*P* < 0.001). Approximately 5 min after the first HBO session, the erythrocytic TBARS concentration did not change in a statistically significant manner compared to the level measured before HBO while after the 14th session, it was increased by 10% (*P* < 0.05). The TBARS concentration in the erythrocytes of the SSNHL patients after the 14th HBO session was 17% lower than that in the control group, and the difference remained statistically significant (*P* < 0.01).

The CAT activity in the erythrocytes of the SSNHL patients before the HBO therapy was 26% higher than that in the control group, and the difference was statistically significant (*P* < 0.001). Approximately 5 minutes after the first HBO session, the CAT activity decreased by 6% (*P* < 0.05) compared to that determined before treatment, while after 14 sessions, it showed a slight increasing trend (*P* > 0.05) compared to that measured after the first session and was nonsignificantly lower than that before the HBO therapy. After both the first and 14th HBO sessions, the CAT activity in the SSNHL patients was significantly higher than that in the control group by 19% (*P* < 0.001) and 22% (*P* < 0.001), respectively.

No statistically significant differences were found in the erythrocytic SOD activity before the HBO therapy in the SSNHL patients and the control group. However, the SOD activity was nonsignificantly lower in the SSNHL patients. Approximately 5 min after the first HBO session, the SOD activity decreased in a statistically nonsignificant manner, while after 14 sessions, it was 7% lower compared to that in the pretreatment level, and the difference was statistically significant (*P* < 0.05). The SOD activity after 14 HBO sessions was 6% lower than that after the first session and 13% lower than that in the control group, and both differences were statistically significant (*P* < 0.05 and *P* < 0.001, respectively).

No statistically significant differences were found in the erythrocytic GPx activity in the SSNHL patients and the control group. However, the GPx activity was nonsignificantly higher in the SSNHL patients than in the control group. Approximately 5 min after the first HBO session, the GPx activity was nonsignificantly (*P* > 0.05) increased compared to the pretreatment value and was significantly higher by 62% (*P* < 0.05) than that in the control group. After 14 HBO sessions, a nonsignificant increasing tendency in the GPx activity compared to that after the first HBO session was observed. The GPx activity at that time point of the study was 28% higher (*P* < 0.05) than that of before the HBO therapy and 73% higher (*P* < 0.001) than that in the control group.

The HGB concentration in the SSNHL patients after the 14th HBO session was 6% lower than that of before the HBO therapy, and the difference was statistically significant (*P* < 0.01). The HCT value determined at that time point was also 6% lower (*P* < 0.01) than that of before treatment.

## 4. Discussion

In this study, no statistically significant changes in the TBARS concentration in the plasma of the SSNHL patients were observed. However, in erythrocytes, the concentration of TBARS after 14 HBO sessions increased compared to the value determined before the HBO therapy, which can indicate an enhanced peroxidation of membrane lipids in these cells. Yet, the erythrocytic TBARS concentration in the SSNHL patients was lower in a statistically significant manner than that in the control group at all time points. Therefore, the observed increase in the TBARS concentration in erythrocytes can also be interpreted as normalisation of redox processes, and the reduced level of TBARS could be a result of intensified antioxidant mechanisms accompanying the oxidative processes occurring in SSNHL. This hypothesis is supported by the significantly higher CAT activity in the SSNHL patients measured before the HBO therapy compared to the control group. Another fact supporting the hypothesis of effective removal of ROS by scavenging mechanisms in the SSNHL patients was also the statistically significant negative correlation between the SOD activity and the TBARS concentration in erythrocytes observed before the HBO therapy (*r* = −0.318; *P* < 0.05) (Table 2, Figure 3).

Despite the proven increase in the generation of ROS in the blood induced by hyperbaric oxygen [14, 15], changes in the levels of TBARS and MDA after HBO therapy reported in the literature are not clear. Both an increase and a decrease in the levels of lipid peroxidation products after this type of treatment have been reported. An increase in, e.g., MDA level in the erythrocytes of divers subjected to hyperbaric exposure was demonstrated by Kozakiewicz et al. [16]. In turn, Benedetti et al. [15] observed an increased level of TBARS in the plasma of patients before their 15th HBO session compared to that of before the first HBO session, with the erythrocytic TBARS concentration showing no significant change. In patients with diabetes mellitus, a statistically significant increase in the MDA concentration in plasma was shown after the first HBO session, while changes observed after the 15th session were not statistically significant [17]. In their study, Paprocki et al. [18] did not demonstrate statistically significant changes in the concentration of TBARS in either the erythrocytes or the plasma of patients subjected to an HBO session, regardless of the fact whether before the experiment, the patients had undergone HBO sessions of no more than 3 times, or more than 23 times. In experimental studies conducted in animals treated with hyperbaric oxygen, as in humans, the observed changes in the concentrations of lipid peroxidation products have varied. A reduction in the concentration of MDA in erythrocytes after HBO therapy compared to the group not treated with HBO has been shown, e.g., in rats with experimentally induced Crohn's disease [19] and with experimentally induced pancreatitis [20]. In turn, an increase in the TBARS concentration has been found in the erythrocytes of rats with streptozotocin- (STZ-) induced diabetes after HBO [21].

Therefore, it seems that the use of HBO generates ROS, but the functioning antioxidant mechanisms protect membrane lipids from excessive peroxidation. Differences reported in various publications can also be associated with the value of pressure at which the HBO sessions are conducted or with the formation of potential adaptive mechanisms with respect to hyperbaric oxygen. It cannot be excluded that the observed differences were affected by the time onset of SSNHL and the initiation of HBO therapy. In this study, HBO therapy was initiated no later than 5 days after the onset of SSNHL, which was in line with the guidelines of the Polish Society of Audiology and Phoniatrics. According to the guidelines, HBO therapy should be used only as supportive treatment during the first two weeks after the onset of SSNHL [1]. However, the effectiveness of HBO therapy in improving hearing is also observed in cases in which this treatment is introduced later, e.g., within 20 days of the onset of hearing loss [22]. Moreover, Topuz et al. [23] demonstrated that HBO therapy increases the effectiveness of conventional therapy when the treatment is started early after the onset of SSNHL.

The level of lipid peroxidation products observed in this study could also be affected by the use of corticosteroids (prednisone) by the patients at a tapered dose. Studies employing experimental models have proven that short-term use of corticosteroids protects various tissues against oxidative damage, but their longer use intensifies lipid peroxidation [24]. In this experiment, the patients took corticosteroids for a short period of time, i.e., up to two weeks. Other studies have also shown that corticosteroids reduce the intensity of lipid peroxidation. Keles et al. [25] demonstrated a decrease in the serum and cerebrospinal fluid concentrations of MDA in patients with multiple sclerosis after corticosteroid therapy. A decrease in lipid hydroperoxide (ROOH) and normalisation of the H_2_O_2_ and TBARS levels have been observed after corticotherapy in Graves' disease patients [26]. The above effects of corticotherapy may be due to the fact that corticosteroids, among other actions, increase the levels of antioxidant enzymes in leukocytes [27] and inhibit the release of superoxide anion by human monocytes [28].

In the study presented in this paper, a statistically significant decrease of 6% (*P* < 0.05) in the CAT activity in the erythrocytes of patients with SSNHL after the first HBO stimulation was observed. After 14 HBO sessions, the CAT activity showed a statistically nonsignificant tendency to increase compared to that determined after the first HBO session. It was higher in a statistically significant manner in the SSNHL patients compared to that in the control group at all time points. In turn, the SOD activity decreased significantly after 14 HBO sessions. It was 7% lower (*P* < 0.05) than that of before the HBO therapy and 6% lower (*P* < 0.05) than that of after the first session. Concurrently, the GPx activity after 14 HBO sessions increased by 26% compared to that measured before the HBO therapy, and the difference was statistically significant (*P* < 0.05). The higher CAT activity in the erythrocytes of the SSNHL patients before the HBO therapy compared to the control group may imply the excessive H_2_O_2_ generation in the course of SSNHL. This was also confirmed by the higher, although statistically nonsignificant, GPx activity in the erythrocytes of the SSNHL patients. Both enzymes are involved in the removal of H_2_O_2_, and erythrocytes are considered as a circulating sink of H_2_O_2_ [29]. Hydrogen peroxide, which is electrically neutral and more stable than superoxide anion, easily passes through biological membranes [5] and, therefore, can migrate from the environment into erythrocytes. Further increase in the GPx activity in erythrocytes to significantly higher values after the 14th HBO session, compared to that measured before the HBO therapy, may indicate potential increase in H_2_O_2_ generation also due to hyperbaric oxygen therapy. Increased H_2_O_2_ generation may be also verified by the statistically significant positive correlation between the activities of GPx and SOD in the erythrocytes of the SSNHL patients after 14 HBO sessions (*r* = 0.356, *P* < 0.05) (Table 2, Figure 4). Hydrogen peroxide can initiate a nonenzymatic degradation of haem, while the products of this degradation initiate oxidative processes in erythrocytes [30].

Paprocki et al. [31], in a preliminary study in patients with SSNHL, demonstrated a reduction of the CAT activity approximately 5 minutes after the completion of a single HBO session. The largest reduction of the CAT activity was observed in patients under 35 years of age. Similarly, in people with different diseases, only the CAT activity decreased approximately 5 min after a single HBO session, but this phenomenon regarded only those patients who had been in HBO sessions no more than 3 times prior to the experiment [18]. In turn, no changes in the CAT activity were observed in people subjected to HBO therapy multiple times (over 23 sessions) before the experiment. The activities of GPx and SOD in the erythrocytes of those patients did not change in a statistically significant manner after the experimental HBO session [18]. No statistically significant changes in the activities of SOD, GPx, and CAT 24 hours after a single HBO session were found in the erythrocytes of healthy people [32]. In another study conducted in healthy people, the GPx activity in erythrocytes increased significantly during HBO therapy, but not after its completion [33]. In studies conducted in animals, changes in the activity of antioxidant enzymes after HBO therapy have not been clear either. For example, an increase in the SOD activity in rapidly contracting muscles and a decrease in the CAT activity in slowly contracting muscles have been observed in rats [34]. Matsunami et al. [35] demonstrated a decrease in the Cu-Zn SOD and CAT gene expression and an increase in the GPx gene expression in all tested organs of rats with experimentally induced diabetes treated with HBO therapy compared to a group of rats with experimentally induced diabetes that were not treated with HBO therapy.

In the SSNHL patients, a statistically significant reduction of haematocrit and haemoglobin after 14 HBO sessions compared to the values measured before the first session was observed. The results obtained by other authors are not definitive. For example, Handy et al. [36] did not demonstrate changes in the haematocrit value and the concentration of haemoglobin in the blood of chronically ill patients with problematic wounds after 20 HBO sessions. In turn, Sinan et al. [37] showed a large reduction in haematocrit in patients after 20 HBO sessions compared to their baseline values, but the difference was not statistically significant. Conversely, a statistically significant decrease in haematocrit and haemoglobin was demonstrated in 16 selected patients after 21 days of HBO therapy [38]. It is possible that long-term, repeated treatment with hyperbaric oxygen affects the process of erythropoiesis, which can be an adaptive mechanism of the body to high pressure and high oxygen concentration.

## 5. Conclusions

SSNHL is accompanied by disturbance in the oxidant-antioxidant equilibrium. Repeated stimulation with hyperbaric oxygen modulates the activity of antioxidant enzymes. It seems that increased generation of hydrogen peroxide is responsible for the changes in the activity of antioxidant barrier enzymes observed after HBO sessions.

## Figures and Tables

**Figure 1:** Inside the hyperbaric chamber at the Mazovian Centre for Hyperbaric Therapy and Wound Treatment in Warsaw, Poland (photograph: J. Paprocki).

**Figure 2:** The hyperbaric chamber at the Mazovian Centre for Hyperbaric Therapy and Wound Treatment in Warsaw, Poland (photograph: J. Paprocki).

**Figure 3:** Linear regression of superoxide dismutase (SOD) activity versus thiobarbituric acid reactive substances (TBARS) concentration in the erythrocytes of SSNHL patients before HBO therapy (*r* = −0.318, *P* < 0.05).

**Figure 4:** Linear regression of superoxide dismutase (SOD) activity versus glutathione peroxidase (GPx) activity in the erythrocytes of SSNHL patients after 14 HBO sessions (*r* = 0.356, *P* < 0.05).

**Table 1:** Markers of oxidative stress in the blood of healthy members of the control group and patients with sudden sensorineural hearing loss (SSNHL) treated with hyperbaric oxygen (HBO) therapy and the values of haemoglobin concentration and haematocrit in the SSNHL patients.

Parameters	Control	SSNHL patients		
		Before HBO therapy	~5 min after first HBO session	After 14 HBO sessions
TBARS in plasma (nmol MDA/mL)	0.38 ± 0.07	0.43±0.10^++^	0.45±0.08^+++^	0.42 ± 0.10^+^
TBARS in erythr. (nmol MDA/g Hb)	32.60 ± 6.77	24.70±8.25^+++^	24.47±8.07^+++^	27.06 ± 8.39^++^^∗^
CAT (10^4^ IU/g Hb)	52.97 ± 6.09	66.64±10.25^+++^	62.93 ± 8.23^+++^^∗^	64.75±10.07^+++^
SOD (U/g Hb)	816.73 ± 128.64	764.44 ± 159.00	757.06 ± 141.50	713.26 ± 72.89^+++^^∗^^†^
GPx (U/g Hb)	5.54 ± 4.05	7.51 ± 4.64	8.97 ± 4.42^+^	9.61 ± 4.75^+++^^∗^
HGB (g/mL)		15.58 ± 1.39		14.64 ± 1.43^∗∗^
HCT (%)		43.88 ± 3.47		41.29 ± 3.60^∗∗^

TBARS: thiobarbituric acid reactive substances; CAT: catalase; GPx: glutathione peroxidase; SOD: superoxide dismutase; HGB: haemoglobin; HCT: haematocrit. The values are expressed as means ± standard deviations (SD) of the means. ^+^Statistically significant difference compared to the control group (^+^*P* < 0.05; ^++^*P* < 0.01; ^+++^*P* < 0.001). ^∗^Statistically significant difference compared to parameters measured before the HBO therapy (^∗^*P* < 0.05; ^∗∗^*P* < 0.01). ^†^Statistically significant difference compared to the parameters measured after the 1st HBO session (^†^*P* < 0.05).

**Table 2:** Statistically significant correlation coefficients between the parameters measured in the patients with SSNHL (studied group).

	Parameters	*r*
Before HBO therapy	TBARS in plasma/SOD	0.458^∗∗^
	TBARS in erythrocytes/SOD	−0.318^∗^
	CAT/GPx	0.395^∗^
~5 min after first	TBARS in plasma/SOD	0.365^∗^
HBO session	CAT/GPx	0.317^∗^
After 14 HBO sessions	SOD/GPx	0.356^∗^

TBARS: thiobarbituric acid reactive substances; CAT: catalase; GPx: glutathione peroxidase; SOD: superoxide dismutase. ^∗^*P* < 0.05. ^∗∗^*P* < 0.01.

## Data Availability

The study data used to support the findings of this study are included within the article.
